# lncRNA-NEAT1 Sponges miR-128 to Promote Inflammatory Reaction and Phenotypic Transformation of Airway Smooth Muscle Cells

**DOI:** 10.1155/2022/7499911

**Published:** 2022-01-17

**Authors:** Danyang Song, Yajing Jiang, Qiuju Zhao, Jinling Li, Yuqi Zhao

**Affiliations:** Department of Pediatric, Cangzhou Central Hospital, Cangzhou, Hebei 061000, China

## Abstract

**Objective:**

Pediatric asthma is still a health threat to the children. Long noncoding RNA-NEAT1 (lncRNA-NEAT1) was reported to be positively correlated with the severity of asthma. We aimed to study the effects and mechanism of lncRNA-NEAT1on inflammatory reaction and phenotypic transformation of airway smooth muscle cells (ASMCs) in the bronchial asthma.

**Method:**

The degree of lncRNA-NEAT1 and miR-128 mRNA in children with bronchial asthma and healthy individuals was tested by qRT-PCR. After the inflammatory reaction and phenotypic transformation of PDGF-BB-induced ASMCs, the expression of lncRNA-NEAT1 or miR-128 in the AMSC was disturbed in the AMSC. Subsequently, the expression of lncRNA-NEAT1 and miR-128 was detected by the way of qRT-PCR, and western blot was applied to measure the expression of MMP-2, MMP-9, *α*-SMA, calponin, NF-*κ*B, and so on in the cells. The content of TNF-*α*, IL-1*β*, IL-6, and IL-8 in the cell culture supernatant was checked by ELISA. MTT, Transwell, and flow cytometry were used to detect cell proliferation, migration, and apoptosis. Further, the targeting relations between lncRNA-NEAT1 and miR-128 were evaluated by the dual-luciferase reporter assay.

**Result:**

In the sputum of children with bronchial asthma, lncRNA-NEAT1 was significantly upregulated while miR-128 was rapidly downregulated. Besides, lncRNA-NEAT1 and miR-128 were competitively combined and, for their expression, negatively correlated.

**Conclusion:**

lncRNA-NEAT1 sponges miR-128 to boost PDGF-BB-induced inflammatory reaction and phenotypic transformation of ASMCs to aggravate the occurrence and development of childhood bronchial asthma.

## 1. Introduction

Bronchial asthma (hereinafter referred to as asthma) is a common chronic airway inflammatory disease of the respiratory system [1], which may cause serious incidence rate and high mortality in the world [2]. The data from the Global Initiative for Asthma (GINA) showed that there were 300 million asthmatics in the world in 2014. The number was anticipated to add to 400 million, including 14% children among them in 2025 [3, 4]. More terribly, children with asthma may have a pattern of rapidly evolving, frequent, and often severe exacerbations [5]. Glucocorticoid is the main choice to make a comprehensive therapy, but long-term use may cause multiple side effects, such as hormone dependence, inhibition of growth in children, and an increase in family pressure and waste of medical resources in the society [6–8]. Therefore, in order to look for potential new medicines, as well as prevent the occurrence and development of asthma fundamentally, a further study on pathogenesis of asthma is important.

According to a traditional view, airway inflammation is the core part of the mechanism of childhood asthma, and airway remodeling is a result of the development of chronic airway inflammation [9, 10]. The stage of airway remodeling is irreversible and will affect the prognosis of asthmatic children [11]. Airway smooth muscle cells (ASMCs) can not only regulate airway relaxation and contraction under the stimulation of inflammation and mechanical strain but also participate in the whole process of airway remodeling in asthma [12, 13]. Evidence suggests that there is a strong regional relationship between airway remodeling and airway inflammation. Under the microenvironment of asthma, a variety of cytokines could stimulate airway smooth muscle cells to turn to a synthetic phenotype [14]. Therefore, inhibition of cytokine secretion and phenotypic transformation of ASMCs may prevent the development of asthma in children.

Long non-coding RNAs (lncRNAs) are a class of endogenous RNAs over 200 nucleotides in length [15–17]. lncRNAs are allowed to join in pathologic progress in all kinds of mechanisms from the level of transcription to the level of posttranscription [18, 19]. lncRNA-NEAT1 (NEAT1 is short for nuclear paraspeckle assembly transcript 1), which is also called VINC, is ranked no. 11 on the chromosome of human. There is evidence that lncRNA-NEAT1 is intricately associated with inflammation and can be used as an inflammatory regulator in human lupus, sepsis, and atherosclerosis [20–22]. lncRNA-NEAT1 has been reported to be associated with the progression of asthma [23]. Airway remodeling involves inflammation, migration, and proliferation [24, 25], which has led to the speculation that lncRNA-NEAT1 has participated in the regulation of gene expression, affecting cell differentiation, migration, and proliferation, leading to the occurrence and development of asthma.

In this study, we determine the expression of lncRNA-NEAT1 in children with asthma, discuss its effect on the level of inflammatory cytokines and phenotypic transformation of PDGF-BB-treated ASMCs, and try to provide a new experimental basis for understanding the pathogenesis of pediatric asthma.

## 2. Materials and Methods

### 2.1. Collection and Treatment of Clinical Samples

After getting permission from the Cangzhou Central Hospital ethical committee (2020-288-02(Y)), we chose 24 children with acute bronchial asthma as the asthma group according to *Guidelines for Diagnosis, Prevention and Treatment of Bronchial Asthma in Children*. The asthma group included 13 males and 11 females (average age: 7.54 ± 2.06 years). Then, 24 healthy children (HC group) were chosen as the control group, including 12 males and 12 females (average age: 7.71 ± 2.03 years). Both children and their parents agreed on this research and had signed consent forms. Then, we induced sputum by hypertonic saline with ultrasonic nebulization for the two groups of children [26]. Forming and viscous sputum was selected and observed by using a microscope; when squamous epithelial cells ≤ 20%, the sputum was qualified [27]. Then, the qualified sputum was treated with 0.1% DTT (Sigma). After centrifugation, the sputum supernatant was kept at -20°C for subsequent tests.

### 2.2. Cell Culture and Cell Membrane Formation

Human ASMCs had been purchased from the Cell Bank of Institute of Basic Medical Sciences, Chinese Academy of Medical Science. The culture conditions were as follows: F12K medium with 10% of fetal bovine serum, 100 U/mL penicillin and 100 *μ*g/mL streptomycin, 37°C, and 5% CO_2_. Then, 0.25% of trypsin was applied to digest AMSC for getting cell suspension to be seeded in the 6-well plate with a density of 2 × 10^5^ cells/well. The PDGF-BB group was given 10 ng/mL PDGF-BB to induce cell activation^,^ while there is no treatment in the blank control group. After 48 h, the state of cells was observed; also, mRNA and protein were collected for the following experiments.

### 2.3. Cell Transfection

The vector carrying lncRNA-NEAT1 interference sequence with its corresponding unloaded sh-NC, sh-NEAT1, and miR-128 inhibitor was synthesized and cloned by Sangon Biotechnology Co., Ltd., which was confirmed by restriction enzyme analysis and sequencing. After that, AMSC in the logarithmic growth phase was seeded into a 12-well plate. When cell confluence came up to 50%-60%, sh-NC, sh-NEAT1, and miR-128 inhibitor were transfected into cells, respectively, according to the instructions of the Lipofectamine 2000 reagent (Thermo Fisher Scientific, America). After 6 h, the original medium was replaced by a new one to culture cells for another 48 h. Finally, the cells were collected for subsequent experiments.

### 2.4. MTT

Treated cells were selected to digest and count. Then, 5000 cells were put into each well in 96-well plates, with 5 parallel wells in each group. After cell adhesion, the cells would be cultured for 1, 2, 3, and 4 days, respectively. Then, the medium was aspirated, and the prepared MTT solution was added into the plates, and then, they were put into an incubator for 4 h. Subsequently, an enzyme-labeling instrument was prepared to measure optical density absorbance of 96-well plates (490 nm). Finally, the cellular growth curve would be plotted, with time as its horizontal scale and optical density absorbance as its vertical scale.

### 2.5. Transwell Assay

Cells in the logarithmic phase were selected to digest and count. These cells were seeded on the Transwell upper chamber (5000 cells/well) containing 200 *μ*L serum-free medium. The lower chamber was added with 600 *μ*L medium containing 20% FBS. After that, the Transwell inserts were cultured in an incubator with 5% CO_2_ at 37°C. The Transwell inserts were fixed with methanol for 15 min and stained with 0.5% crystal violet for 20 min. Then, the cells in the upper chamber were wiped off. After ten fields of view were randomly selected, cells beneath the polycarbonate film were photographed in order to count and conduct a statistical analysis.

### 2.6. Apoptosis

Cells were collected and counted. Further, 50000-100,000 cells were centrifuged at 1000 r/min for 5 minutes, and then, the supernatant was aspirated. Subsequently, Annexin V-FITC binding solution 195 *μ*L was added into these cells to resuspend gently. After that, 5 *μ*L Annexin V-FITC reagent was added and mixed gently. It was put under light-avoided condition for ten minutes at ambient temperature. Then, 200 *μ*L Annexin V-FITC binding solution was added and resuspended gently. According to the result of testing samples, Annexin V-FITC combined with flow cytometry showed green while the PI showed red. Further analysis was conducted based on the result.

### 2.7. ELISA

The treated cell supernatant was collected to detect the release levels of TNF-*α*, IL-1*β*, IL-6, and IL-8 according to the corresponding instructions of detection kits, respectively (R&D Systems). According to the standard curve, the concentrations of TNF-*α*, IL-1*β*, IL-6, and IL-8 were calculated.

### 2.8. qRT-PCR

The Trizol reagent was used to extract fresh frozen tissues or cellular total RNA. Then, a cDNA transcription kit was applied to reverse transcribe 500 ng RNA into cDNA with the following conditions: 30 minutes at 16°C for transcription, 30 minutes at 42°C for incubation, and 5 min at 85°C for enzymatic inactivity. We made a quick quantification using SYBRH Select Master Mix (Invitrogen). The following parameters were prepared for a transcription reaction: 30 minutes at 16°C, 30 minutes at 42°C, and 5 minutes at 84°C. The following parameters of qRT-PCR reaction were used: 2 minutes at 95°C, 15 s at 95°C, and 15 s at 60°C for a total of 40 cycles. All results were standardized by GAPDH expression. And the 2^−ΔΔCt^ method was utilized for quantitative analysis. The primers used were as follows: lncRNA-NEAT: 5′-CGCCGATATTGGTCGGATGAT-3′ and 5′-TTCAGCGTACACCTAATCGGTATG-3′; GAPDH: 5′-AACGGATTTGGTCGTATTG-3′ and 5′-GGAAGATGGTGATGGGATT-3′; miR-128: 5′-CGCCGATATTGGTCGGATGAT-3′ and 5′-TTCAGCGTACACCTAATCGGTATG-3′; and U6: 5′-CCGTCGTAGGCAGCCTCTACGCT-3′ and 5′-GCATCCAACGTACGCTCATCGT-3′.

### 2.9. Western Blot

After each group cells were extracted, RIPA lysis solution with 1% PMSF was added and mixed. Then, the supernatant was collected when centrifugation of the mixture was finished at 4°C (10000 × *g*). BCA kits (Thermo Fisher Scientific, America) were applied for protein quantification. With the temperature heated to 100°C, total protein electrophoresis was conducted for a 5-minute incubation. SDS-PAGE was followed by protein transfer to PVDF membranes, and then, a blocking step utilizing 5% TBS was conducted. After that, at 4°C, the membranes were incubated with primary antibodies, rabbit monoclonal antibody MMP-2 (1 : 1000, ab92536), rabbit monoclonal antibody MMP-9 (1 : 1000, ab76003), mouse monoclonal antibody *α*-SMA (1 : 1000, ab5831), rabbit monoclonal antibody calponin (1 : 1000, ab46794), rabbit monoclonal antibody NF-*κ*Bp65 (1 : 1000, ab32536), rabbit monoclonal antibody IKK*β* (1 : 1500, ab124957), rabbit monoclonal antibody I*κ*B*α* (1 : 1000, ab32518), and rabbit monoclonal antibody GAPDH (1 : 1000, ab181602) for a night. On the second day, the products of incubation were taken out and washed for three times. Then, membranes were incubated with a secondary antibody, horseradish peroxidase-coupled polyclonal goat anti-rabbit IgG (1 : 1000, ab6721), at ambient temperature for one hour and then were washed for times. The chemiluminescence of membranes was enhanced so the results could be analyzed by using the X-ray film imaging system. Then, the image was quantitatively determined by using ImageJ (NIH).

### 2.10. Dual-Luciferase Reporter Assay

During this section, wild-type or mutant plasmids with lncRNA-NEAT1 3′-UTR were built; then, the Lipofectamine 2000 reagent (Semerfeld, USA) was utilized to cotransfect the plasmids with miR-128 mimics or NC into ASMCs. The luciferase activities of the 4 groups were checked, respectively, by using the dual-luciferase reporter assay system (Promega).

### 2.11. Statistical Analysis

All the experiments were carried out in triplicate. The results were statistically analyzed by using SPSS 22.0. Measurement data was expressed as mean ± standard deviation (SD). Comparison between two groups was conducted by the *t*-test, while comparison among multigroups was performed by one-way ANOVA. Each experiment was repeated three times at least. A statistically significant difference could be suggested if *P* < 0.05.

## 3. Result

### 3.1. Differential Expression of lncRNA-NEAT1 for the Sputum of Children with Asthma

Firstly, qRT-PCR was applied to test the expression of lncRNA-NEAT1 in the sputum of children with asthma. The result confirmed that, compared with the HC group, lncRNA-NEAT1 expression in the asthma group increased significantly (Figure 1).

### 3.2. Downregulation of lncRNA-NEAT1 Suppresses the PDGF-BB-Induced Proliferation, Migration, and Phenotype Transformation in ASMC

PDGF-BB was applied to induce the phenotypic transformation of ASMCs. Figure 1(a) shows that, compared with the control group, PDGF-BB stimulation significantly increased the expression of lncRNA-NEAT1. For the exploration of the role of lncRNA-NEAT1 in ASMCs, we transfected ASMCs with sh-NEAT1 or sh-NC and generated lncRNA-NEAT1-knockdown ASMCs confirmed by RT-PCR (Figure 1(a)). Compared with the control group, PDGF-BB treatment significantly induced ASMC proliferation and migration. After knocking down lncRNA-NEAT1 expression, the abilities to proliferate and migrate were observed (Figures 2(b)–2(d)). The western blot assay showed that PDGF-BB treatment significantly increased the expression of MMP-2 and MMP-9 proteins, while it decreased the expression of MMP-2 and MMP-9 proteins of ASMCs in comparison with the control group, and these effects were markedly reversed by lncRNA-NEAT1 knockdown (Figures 2(e) and 2(f)).

### 3.3. Downregulation of lncRNA-NEAT1 Suppresses the PDGF-BB-Interfered Expression of Inflammatory Factors in ASMC

Further detection was made to ensure the effect of lncRNA-NEAT1 expression on inflammatory factors in AMSCs. According to the results of ELISA, compared with the control group, the content of TNF-*α*, IL-1*β*, IL-6, and IL-8 in the cell culture supernatant in the PDGF-BB group increased significantly. After interfering with lncRNA-NEAT1 expression, the release level of TNF-*α*, IL-1*β*, IL-6, and IL-8 reduced quickly (Figures 3(a)–3(d)).

### 3.4. lncRNA-NEAT1 Targets miR-128 in ASMC

A further research was made to explore the function mechanism of lncRNA-NEAT1 on asthma. Firstly, the target gene of lncRNA-NEAT1 was predicted by using Starbase V2.0 (http://starbase.sysu.edu.cn/), and obvious binding sites were found between lncRNA-NEAT1 and miR-128. The dual-luciferase reporter assay was used to identify the binding between lncRNA-NEAT1 and miR-128. The result showed that cotransfection of miR-128 mimics and lncRNA-NEAT1-wt can significantly reduce the intensity of luciferase in ASMCs (Figure 4(a)). Besides, low expressions of miR-128 were also found in asthmatic children (Figure 4(b)). And according to qRT-PCR detection, low expressions of miR-128 were also found in the PDGF-BB group while after suppressing lncRNA-NEAT1, the expression of miR-128 increased significantly (Figure 4(c)). Correlation analysis also suggested that lncRNA-NEAT1 and miR-128 were correlated negatively. It indicated that lncRNA-NEAT1 could combine with miR-128 competitively (Figure 4(d)).

### 3.5. Downregulation of lncRNA-NEAT1 Can Interfere with Promoting Effects of miR-128 on the Proliferation, Migration, Phenotype Transformation, and Inflammatory Reaction in PDGF-BB-Induced ASMC

In order to explore whether lncRNA-NEAT1 played its biology function by controlling miR-128, we used PDGF-BB to induce inflammatory reaction and phenotypic transformation of AMSCs, and then, ASMCs were transfected with the miR-128 inhibitor or sh-NEAT1+miR-128 inhibitor.

The results suggested that the miR-128 inhibitor significantly increased the cell proliferation rate and migration ability in comparison with the PDGF-BB group, and these effects were markedly reversed by lncRNA-NEAT1 knockdown (Figures 5(a)–5(c)). Compared with the PDGF-BB group, the expression of MMP-2 and MMP-9 proteins was significantly increased, and the expression of *α*-SMA and calponin proteins was significantly reduced in the PDGF-BB+miR-128 inhibitor group (Figures 6(a)–6(b)). lncRNA-NEAT1 knockdown can reverse the expression level of MMP-2, MMP-9, *α*-SMA, and calponin proteins (Figures 6(a) and 6(b)). Results identified that the miR-128 inhibitor significantly rose up the release ability of TNF-*α*, IL-1*β*, IL-6, and IL-8 in ASMCs, while this enhancement was significantly reversed by lncRNA-NEAT1 knockdown (Figures 6(c)–6(f)).

### 3.6. lncRNA-NEAT1 Activates the NF-*κ*B Signaling Pathway in ASMC with Induction of PDGF-BB

To investigate whether lncRNA-NEAT1 played its biological function by the NF-*κ*B signaling pathway, we used a western blot assay to detect the expression levels of NF-*κ*Bp65, IKK*β*, and I*κ*B*α* in ASMCs. The results suggested that PDGF-BB treatment significantly increased the expression levels of NF-*κ*Bp65 and IKK*β* in ASMCs and decreased the expression level of I*κ*B*α*. Compared with the PDGF-BB+shNC group, NEAT1 knockdown prevented the increase in the expression of NF-*κ*Bp65 and IKK*β* and promoted the expression of I*κ*B*α* (Figure 7(a)). Subsequently, ASMCs were treated with PDTC to inhibit the NF-*κ*B signaling pathway. We observed that PDTC treatment inhibited the expression of NF-*κ*Bp65 and IKK*β* and increased the expression level of I*κ*B*α*; on this basis, lncRNA-NEAT1 knockdown could further inhibit the NF-*κ*B signaling pathway (Figure 7(b)).

## 4. Discussion

Pediatric asthma, with a prevalence rate at 5-10%, is a common disease during childhood and adolescence. The prevalence of asthma in children (0-17 years old) has risen up from 3.5% to 9.5% in 30 years [28, 29]. A lot of lncRNAs have been verified to have important influence on respiratory diseases [30, 31]. The abnormal expression of lncRNA-MALAT1 [32], lncRNA-COX2 [33], linc-MAF-4 [34], and other lncRNAs has been applied as prognostic markers for various lung diseases. More and more evidences show that lncRNA-NEAT1 is involved in the pathogenesis of asthma. lncRNA-Neat1 has been reported to promote the level of inflammatory cytokines in ASMCs through the miR-139/JAK3/STAT5 signaling network [35]. lncRNA-NEAT1 negatively regulates miR-200a/b to aggravate the inflammatory response of asthma [36]. In the experiment, it is proven that the expression of lncRNA-NEAT1 is high in the sputum of children with asthma.

Airway remodeling is one of the important features of childhood asthma [37]. The proliferation and migration of ASMCs will lead to thickening of the airway wall, which in turn will participate in the development of airway remodeling in asthma [38]. Previous studies have shown that the levels of MMP-2 and MMP-9 around the inflamed airways of asthmatic mice are significantly increased [39]. Cheng et al. reported that ABCA1 can inhibit the migration ability of rat ASMCs and reduce the mRNA levels of MMP-2 and MMP-9 [40].

AMSC phenotypic regulation is defined as a reversible transition between the contractile phenotype and proliferative phenotype [41]. *α*-Smooth actin (*α*-SMA) is the main marker of smooth muscle, reflecting the alterations in the numbers and contraction ability of smooth muscle. Fibroblasts that express *α*-SMA can result in luminal stenosis in shrinkage. Most studies found that myofibroblasts could facilitate the deposition of type I and III collagens and lead to the reconstruction of the extracellular matrix and then could cause vascular wall thickening and stiffness [42, 43]. *α*-SMA and type I collagen were reported to be important indexes in early airway remodeling. It is reported that PDGF-BB can promote the proliferation and migration of ASMCs, mimicking the cellular state of children with asthma [44–46]. The results indicated that downregulation of lncRNA-NEAT1 could inhibit PDGF-BB-induced migration and phenotype conversion in ASMCs.

MicroRNAs (miRNAs), a class of small noncoding RNAs comprising 19–25 nucleotides, can inhibit gene expression at the posttranscriptional level. In recent years, more and more evidences have shown that lncRNAs can work by a ceRNA mechanism, competitively binding with miRNAs to affect the silencing of downstream target genes by miRNAs. We identified the interaction between miR-128 and lncRNA-NEAT1 through the bioinformatics prediction and dual-luciferase reporter assay. miR-128 has been shown to reduce the radioresistance of glioma stem-like cells by coordinately targeting PRC [47]. Song et al. demonstrated that miR-128 inhibits cigarette smoke-induced inflammatory response in mice with chronic obstructive pulmonary disease. miR-128 inhibits apoptosis and inflammation of pulmonary microvascular cells induced by cigarette smoke extract by downregulating BRD4 [48]. It is reported that miR-128 is significantly downregulated in the serum of asthmatic horses [49]. We found that miR-128 is downregulated in the sputum of children with asthma. Silencing lncRNA-NEAT1 significantly reversed the effect of miR-128 knockdown on PDGF-BB-induced ASMC phenotypic transition and inflammation. The above results suggest that the activity of miR-128 is required to inhibit PDGF-BB-stimulated ASMC phenotypic transition and inflammatory response induced by lncRNA-NEAT1 knockdown.

NF-*κ*B is an important nuclear factor that widely existed in multiple tissues and cells, which can participate in various biological activities, such as immune response, inflammatory response, apoptosis, and tumorigenesis. The NF-*κ*B signaling pathway is a classic pathway involved in the pathogenesis of asthma and various pathological changes, such as airway hyperresponsiveness, airway inflammation, and airway remodeling [50–52]. By previous studies, our group has found that asthma airway smooth muscle can transfer from being synthetic to contractile by interfering with the NF-*κ*B signaling pathway [53]. Kong et al. [52] found that PDGF-BB stimulation can significantly increase the expression levels of inflammatory factors TNF-*α*, IL-1*β*, IL-6, and IL-8 in ASMCs. YiQi GuBen pretreatment can significantly improve the inflammatory response of PDGF-BB-treated ASMCs by inhibiting the NF-*κ*B signaling pathway. In this study, we found that lncRNA-NEAT1 knockdown significantly reduced the expression of NF-*κ*Bp65 and IKK*β*, increased the expression of I*κ*B*α*, and decreased the levels of TNF-*α*, IL-1*β*, IL-6, and IL-8 in PDGF-BB-treated ASMCs.

## 5. Conclusion

In conclusion, according to this research, the expression of lncRNA-NEAT1 is high in children patients' sputum. The mechanism may occur at the following order: with lncRNA-NEAT1 binding to miR-128 competitively, the signaling pathway of NF-*κ*B is activated, and after that, PDGF-BB-induced inflammatory reaction and phenotype conversion of ASMCs are promoted; then, childhood asthma is aggravated. It is suggested that lncRNA-NEAT1/miR-128 can be applied as a biomarker to cure childhood asthma, which offers a new way to the early diagnosis and treatment of the disease. However, there were any animal models to verify results in this paper. In subsequent study, more reliable theoretical basis and experimental data will be offered to make lncRNA-NEAT1/miR-128 a prognostic marker of childhood asthma by researching clinical samples and animal models of asthma diseases.

## Figures and Tables

**Figure 1:** Expression of lncRNA-NEAT1 in the sputum of children with asthma. ^∗∗^*P* < 0.01*vs.* HC group.

**Figure 2:** Effects of declining lncRNA-NEAT1 on the PDGF-BB-induced proliferation, migration, and phenotype transformation in ASMC. (a) qRT-PCR was used to detect lncRNA-NEAT1 expression in the groups of ASMC after induction of PDGF-BB. (b) MTT was utilized to measure cell viability in the groups of ASMCs in different times. (c) MTT was used to detect cell proliferation in the groups of ASMCs in different times. (d) Transwell was applied to detect cell migration ability in the groups of ASMCs. (e) Western blot was used to measure the expression of MMP-2 and MMP-9 related to proliferation and migration. (f) Western blot was utilized to detect the expression of *α*-SMA and calponin proteins related to phenotypic transformation. ^∗∗^*P* < 0.01*vs.* control; ^##^*P* < 0.01*vs.* PDGF-BB+sh-NC. The values were presented as mean ± SD (*n* = 3).

**Figure 3:** Effects of declining lncRNA-NEAT1 on the expression of ASMC inflammatory factors interfered with PDGF-BB. (a–d) ELISA was utilized to detect TNF-*α* level (a), IL-1*β* level (b), IL-6 level (c), and IL-8 level (d) in the ASMC supernatant of medium in groups. ^∗∗^*P* < 0.01*vs.* control group; ^##^*P* < 0.01*vs.* PDGF-BB+sh-NC group. The values were presented as mean ± SD (*n* = 3).

**Figure 4:** Connection between lncRNA-NEAT1 and miR-128 expression. (a) Starbase V2.0 was used to predict the target gene of lncRNA-NEAT1, and the dual-luciferase reporter assay verified that lncRNA-NEAT1 targeted miR-128. ^∗∗^*P* < 0.01*vs.* NC mimic group. (b) qRT-PCR was adopted for measuring the miR-128 expression in the sputum of children with asthma and children with health examination. ^∗∗^*P* < 0.01*vs.* HC group. (c) qRT-PCR was utilized to measure the expression level of miR-128 in ASMCs. ^∗∗^*P* < 0.01*vs.* control group; ^##^*P* < 0.01*vs.* PDGF-BB+sh-NC group. (d) Correlation analysis of the relations between miR-128 and lncRNA-NEAT1. The values were presented as mean ± SD (*n* = 3).

**Figure 5:** Downregulation of lncRNA-NEAT1 affects the effects of miR-128 inhibitor on PDGF-BB-induced proliferation and migration in ASMC. (a) MTT was applied to detect the cell viability in ASMCs in different times. (b) MTT was used to measure the cell viability in ASMCs. (c) Transwell was utilized to detect cell migration ability in ASMCs. ^∗∗^*P* < 0.01*vs.* PDGF-BB group, ^##^*P* < 0.01*vs.* PDGF-BB+miR-128 inhibitor group. The values were presented as mean ± SD (*n* = 3).

**Figure 6:** Effects of downregulation of lncRNA-NEAT1 on the phenotype transformation and inflammatory response of PDGF-BB-induced ASMC by the miR-128 inhibitor. (a) Western blot was used to measure the expression levels of MMP-2 and MMP-9 proteins related to proliferation and migration, (b) Western blot was utilized to detect the expression levels of *α*-SMA and calponin proteins related to phenotypic transformation. (c) ELISA was applied to check the release level of TNF-*α* in the culture supernatant of ASMCs from each group. (d) ELISA was applied to test the release level of IL-1*β* in the culture supernatant of ASMCs from each group. (e) ELISA was applied to test the release level of IL-6 in the culture supernatant of ASMCs from each group. (f) ELISA was applied to test the release level of IL-8 in the culture supernatant of ASMCs from each group. ^∗∗^*P* < 0.01*vs.* PDGF-BB group; ^##^*P* < 0.01*vs.* PDGF-BB+miR-128 inhibitor group. The values were presented as mean ± SD (*n* = 3).

**Figure 7:** Effects of lncRNA-NEAT1 on the NF-*κ*B signaling pathway in ASMC induced by PDGF-BB. (a) Western blot was used to measure the expression levels of NF-*κ*Bp65, IKK*β*, and I*κ*B*α* proteins in the control group, PDGF-BB group, PDGF-BB+shNC group, and PDGF-BB+sh-NEAT1 group. ^∗∗^*P* < 0.01*vs.* control group; ^##^*P* < 0.01*vs.* PDGF-BB+shNC group. (b) Western blot was used to measure the expression levels of NF-*κ*Bp65, IKK*β*, and I*κ*B*α* proteins in PDGF-BB-induced ASMC that was transfected with sh-NEAT1 and sh-NEAT1+PDTC. ^∗∗^*P* < 0.01*vs.* PDGF-BB group; ^##^*P* < 0.01*vs.* PDGF-BB+PDTC group. The values were presented as mean ± SD (*n* = 3).

## Data Availability

The data used to support the findings of this study are available from the corresponding author upon request.
